This article has been retracted.

# Genetic causal relationship between gut microbiota and basal cell carcinoma: A two‐sample mendelian randomization study

**DOI:** 10.1111/srt.13804

**Published:** 2024-06-19

**Authors:** Pan Luo, Dejin Gao, Qingguo Zhang

**Affiliations:** ^1^ Department of Comprehensive Plastic Surgery Plastic Surgery Hospital Chinese Academy of Medical Sciences and Peking Union Medical College Beijing China

**Keywords:** basal cell carcinoma, causality, genetics, gut microbiota, mendelian randomisation study

## Abstract

**Objective:**

Research has previously established connections between the intestinal microbiome and the progression of some cancers. However, there is a noticeable gap in the literature in regard to using Mendelian randomisation (MR) to delve into potential causal relationships between the gut microbiota (GM) and basal cell carcinoma (BCC). Therefore, the purpose of our study was to use MR to explore the causal relationship between four kinds of GM (Bacteroides, Streptococcus, Proteobacteria and Lachnospiraceae) and BCC.

**Methods:**

We used genome‐wide association study (GWAS) data and MR to explore the causal relationship between four kinds of GM and BCC. This study primarily employed the random effect inverse variance weighted (IVW) model for analysis, as complemented by additional methods including the simple mode, weighted median, weighted mode and MR‒Egger methods. We used heterogeneity and horizontal multiplicity to judge the reliability of each analysis. MR‐PRESSO was mainly used to detect and correct outliers.

**Results:**

The random‐effects IVW results showed that Bacteroides (OR = 0.936, 95% CI = 0.787–1.113, *p* = 0.455), Streptococcus (OR = 0.974, 95% CI = 0.875–1.083, *p* = 0.629), Proteobacteria (OR = 1.113, 95% CI = 0.977–1.267, *p* = 0.106) and Lachnospiraceae (OR = 1.027, 95% CI = 0.899–1.173, *p* = 0.688) had no genetic causal relationship with BCC. All analyses revealed no horizontal pleiotropy, heterogeneity or outliers.

**Conclusion:**

We found that Bacteroides, Streptococcus, Proteobacteria and Lachnospiraceae do not increase the incidence of BCC at the genetic level, which provides new insight for the study of GM and BCC.

## 1 INTRODUCTION

Basal cell carcinoma (BCC) ranks as the most prevalent skin cancer type and is a predominant cancer in humans, particularly among the older population.^1^ Ultraviolet radiation (UVR), ionising radiation, arsenic exposure, immunosuppression and organ transplantation are considered to be potential risk factors for BCC. Ultraviolet radiation is directly related to the occurrence of basal cell carcinoma because ultraviolet radiation can damage DNA and induce mutations in tumour‐suppressor genes.^2^ The onset of basal cell carcinoma likely arises from intricate interplay among environmental, phenotypic and genetic determinants.^3^ The incidence of BCC in the United States is estimated to reach 4.3 million cases per year. The high incidence of BCC brings an enormous public health economic burden.^4^

The human gut hosts approximately 100 trillion microbes, a number that is tenfold the count of eukaryotic cells in the human body, representing 1.5–2 kg of an individual's weight.^5^ Shifts in the gut microbiota (GM) can manifest through variations in composition (dysbiosis), functionality, or interactions between the microbiota and host, and these changes have direct links with multiple diseases.^6^ Microbial disorders may lead to many diseases, including cancer.^7^ For instance, the gut flora influences several gastrointestinal (GI) cancers, encompassing those of the oesophagus, stomach, colon, liver and pancreas.^8^ Moreover, research indicates that the intestinal microbiome facilitates the onset and progression of lung cancer through modulation of metabolic pathways, suppression of immune cell activity, and generation of proinflammatory agents.^9^ However, no research has explored whether GM has an impact on BCC.

Observational epidemiological studies are prone to confusion, causal reversal and various biases that lead to unreliable causality. Mendelian randomisation (MR) leverages genetic variations as instrumental variables (IV) to probe the causal link between exposure and outcome. Given that genetic variables adhere to Mendel's law of random assortment, they proficiently sidestep confounders and reverse causation issues.^10^, ^11^ Many scientists have employed MR to examine causative connections between GM and multiple illnesses. For example, Long et al. utilised the MR approach to study the link between the gut microbiota and several cancers, including breast, colorectal, ovarian, head and neck, lung, endometrial and prostate cancers.^12^ Moreover, Du et al. found no causal relationship between psoriasis and bladder cancer through MR analysis.^13^ However, no studies have utilised MR to probe the causal relationship between GM and BCC. Given this gap, our research sought to utilise the MR technique to examine causality between four specific GM types—Streptococcus, Bacteroides, Proteobacteria and Lachnospiraceae—and BCC.

## 2 METHODOLOGY AND RESOURCES

### 2.1 Research framework

To ascertain whether Bacteroides, Streptococcus, Proteobacteria and Lachnospiraceae exert an influence on basal cell carcinoma, we conducted a two‐sample MR analysis. In this analysis, Streptococcus, Bacteroides, Lachnospiraceae and Proteobacteria served as the exposure variables, whereas basal cell carcinoma was the outcome variable, as depicted in Figure 1. Three suppositions were met by MR analysis: (1) SNPs are strongly related to exposure; (2) SNPs show no association with confounding factors; and (3) SNPs exhibit no direct connection with the outcome and are solely susceptible to the influence of the exposure. All the data utilised in this study were obtained from publicly accessible shared databases. The hypothesis put forth is that there is no causal relationship between the exposures (Bacteroides, Streptococcus, Proteobacteria and Lachnospiraceae) and the outcome (basal cell carcinoma).

**FIGURE 1:** Flowchart of the study.

### 2.2 Data sources

In this research, we procured data on genetic variants associated with Bacteroides, Streptococcus, Proteobacteria and Lachnospiraceae from a comprehensive genome‐wide association study (GWAS). The MiBioGen consortium, which aimed to understand how host genetics may influence the composition of the gut microbiome, systematically collected and thoroughly analysed genome‐wide genotypes in conjunction with 16S faecal microbiome data. This extensive dataset encompasses 18 340 individuals participating in 24 distinct cohorts. The methodologies, encompassing quality control, phenotype processing, and signal selection, have been extensively detailed in previously published research.^14^

For our investigation, we utilised basal cell carcinoma (BCC) data extracted from a detailed GWAS.^15^ This specific study involved extensive GWAS analysis with a sample comprising 17 416 cases and 375 455 controls. In more detail, the research team incorporated multiomics data from a wide range of population‐based genetic studies. This encompassed various data elements, such as expression quantitative trait loci specific to both blood and skin, as well as methylation quantitative trait loci. Through this rigorous process, they identified a set of functionally significant potential BCC susceptibility genes related to their GWAS loci.^15^

### 2.3 Genetic variants

The selection of SNPs related to Bacteroides, Streptococcus, Proteobacteria and Lachnospiraceae was based on GWAS analysis.^16^ The data used in the analysis were obtained from a database provided by the GWAS. First, we selected exposure‐related SNPs at genome‐wide significance (*p*  <  5 × 10−8) as instrumental variables in secondary analysis to maximise specificity. Second, we ensured that none of the SNPs involved in coverage were in strong association with disequilibrium (LD), as LD can lead to skewed results. The samples selected in the analysis process are European samples of the 1000 Genomes Project, and these samples were aggregated (R2 < 0.001) to estimate the LD of SNPs, which can also eliminate undetected SNPs. Then, we manually checked and eliminated all identified SNPs associated with confounders. We used the phenoscanner GWAS database to rule out confounders associated with factors, such as ultraviolet exposure, ionizing radiation, arsenic exposure, immunosuppression and organ transplantation, that can cause basal cell carcinoma. Furthermore, we stipulated a significant number of bases between the two SNPs for our study. Quality control measures were implemented, ensuring that the minor allele frequency was greater than 1%, by using the CEU population's reference data obtained from the renowned 1000 Genomes Project.^17^

These selected SNPs were regarded as IVs for relevant two‐sample MR analysis. Using the R2 value, we estimated how much of the variance in testosterone and oestradiol was explained by each SNP,^18^ with each SNP's instrument strength being evaluated using the F‐statistic^19^ (calculated as $\;F\;=\frac{R^{2}}{1-R^{2}}\;\times \frac{N-K-1}{K}$, $R^{2}=2\times MAF\times \left(1-MAF\right)\times {\left(\frac{\beta }{sd}\right)}^{2}$). The SNPs were eliminated for being palindromic with allele frequencies.^20^ Detailed information can be seen in Tables S1‐S4.

### 2.4 Mendelian randomization analysis

In our research, the primary analytical approach employed was the random effect IVW model. In addition, we utilised associated methods, including the weighted median method,^21^ simple mode method,^22^, ^23^ weighted mode method^22^, ^24^ and MR–Egger method.^25^, ^26^ The IVW model offers dependable causal estimations, especially in scenarios in which horizontal pleiotropy is not present.^27^, ^28^ In the course of the study, considering the influence of heterogeneity and pleiotropic factors, the reference result is the result of random effect IVW. The weighted median method was employed for accurate estimation, utilizing instrumental variables that exhibit an effectiveness rate of at least 50%.^22^ In the given circumstance that the maximum group IV with consistent MR estimation was found to be valid, the causal relationship was estimated by the consistent method based on the weighted mode.^24^ The MR‒Egger model can be used to identify pleiotropy (*p* < 0.05).^29^ However, the estimation accuracy of this method is not high.^30^

### 2.5 Pleiotropy and sensitivity analysis

For the study, the MR‒Egger method was applied to assess the validity of IVs. The intercept term of this model can reflect whether the results of multiple MR analysis are affected by multiple validity factors.^31^ MR‐PRESSO was mainly used to detect and correct outliers. This technique primarily aims to eliminate SNPs that introduce excessive heterogeneity during the analysis, enhancing the estimation precision and minimizing the negative impacts of heterogeneity. When regression analysis was carried out by the MR‒Egger model, the heterogeneity was tested by the Cochran Q method, and its level was determined. A *p* value below 0.05 signified significant heterogeneity in this analysis. To analyse potentially influential SNPs, the leave‐one‐out test was also carried out during the study.

The beta value and OR reflect the association type of exposure and outcome variables. In the primary analysis, a Bonferroni‐corrected *p* value threshold of 0.0125, accounting for four exposures, was employed to denote statistical significance. For all sensitivity analyses, a *p* value threshold of 0.05 was utilised. These analyses were conducted using the TwoSampleMR modules and R version 4.2.2.^32^

## 3 RESULTS

### 3.1 Causal association of bacteroides with basal cell carcinoma

Table 1 shows that no causal link between Bacteroides and basal cell carcinoma based on several MR analysis techniques was found, with IVW showing an OR of 0.936 and a 95% CI between 0.787 and 1.113 (*p* value of 0.455). The *p* values for the weighted median, MR–Egger, weighted mode and simple mode all exceeded 0.05, as illustrated in both Table 1 and Figure 2. Figures S1 and S2 provide detailed visual representations: S1 displays a forest plot illustrating variant‐specific inverse variance estimates, and S2 indicates robust results from a leave‐one‐out test. The funnel plot, depicted in Figure S3, further explores the causal connection between Bacteroides and basal cell carcinoma.

**TABLE 1:** Mendelian randomization results of basal cell carcinoma and gut microbiome.

Exposure	Outcome	Method	SNP(*n*)	Beta	SE	OR (95% CI)	*p* value
Bacteroides	Basal cell carcinoma						
		MR Egger	8	0.341	0.446	1.407(0.586–3.374)	0.473
		Weighted median	8	−0.077	0.102	0.925(0.756–1.131)	0.450
		Inverse variance weighted	8	−0.065	0.088	0.936(0.787–1.113)	0.455
		Simple mode	8	−0.101	0.157	0.903(0.663–1.231)	0.542
		Weighted mode	8	−0.095	0.141	0.909(0.689–1.199)	0.521
Streptococcus	Basal cell carcinoma						
		MR Egger	14	−0.047	0.196	0.953(0.648–1.402)	0.814
		Weighted median	14	−0.008	0.069	0.991(0.864–1.136)	0.899
		Inverse variance weighted	14	−0.026	0.054	0.974(0.875–1.083)	0.629
		Simple mode	14	−0.034	0.121	0.965(0.761–1.224)	0.779
		Weighted mode	14	−0.040	0.113	0.959(0.768–1.199)	0.723
Proteobacteria	Basal cell carcinoma						
		MR Egger	11	0.106	0.199	1.111(0.752–1.643)	0.607
		Weighted median	11	0.115	0.090	1.122(0.939–1.341)	0.203
		Inverse variance weighted	11	0.107	0.066	1.113(0.977–1.267)	0.106
		Simple mode	11	0.180	0.145	1.197(0.899–1.593)	0.244
		Weighted mode	11	0.169	0.151	1.184(0.879–1.594)	0.291
Lachnospiraceae	Basal cell carcinoma						
		MR Egger	16	0.014	0.169	1.014(0.727–1.415)	0.933
		Weighted median	16	−0.008	0.071	0.991(0.861–1.140)	0.901
		Inverse variance weighted	16	0.027	0.067	1.027(0.899–1.173)	0.688
		Simple mode	16	−0.049	0.118	0.951(0.754–1.200)	0.682
		Weighted mode	16	−0.030	0.102	0.969(0.793–1.185)	0.768

**FIGURE 2:** Scatter plot of the causal association between Bacteroides and basal cell carcinoma.

As shown in Table 2, there was no indication of pleiotropy for the relationship between Bacteroides and basal cell carcinoma [odds (intercept), −0.026; *p* = 0.387]. MR‐PRESSO analysis showed no outliers (MR‐PRESSO global *p* value = 0.443). The *p* value from Cochran's Q test suggests the absence of heterogeneity in the analysis, with a Q statistic of 8.060 and a *p* value of 0.233.

**TABLE 2:** Heterogeneity tests and MR‐Egger intercept of gut microbiome causally linked to basal cell carcinoma.

Exposure	Outcome	Egger intercept	*p*‐value^a^	Q‐statistic	Q‐df	*p*‐value^b^	MR‐PRESSO	*p*‐value^c^
Bacteroides	Basal cell carcinoma	−0.026	0.387	8.060	6	0.233	11.660	0.443
Streptococcus	Basal cell carcinoma	0.001	0.912	5.136	12	0.953	11.814	0.807
Proteobacteria	Basal cell carcinoma	6.92e‐5	0.995	6.975	9	0.639	11.224	0.654
Lachnospiraceae	Basal cell carcinoma	9e‐4	0.935	26.001	14	0.125	29.327	0.150

^a^ *p*‐value: MR‐Egger *p*‐value.

^b^ *p*‐value: Cochran's Q test *p*‐value.

^c^ *p*‐value: MR‐PRESSO global *p*‐value.

### 3.2 Causal association of streptococcus with basal cell carcinoma

The outcomes presented in Table 1, specifically the results obtained from IVW and weighted mode, signify the absence of a causal link between Streptococcus and basal cell carcinoma. Streptococcus, as indicated by IVW, exhibited no impact on basal cell carcinoma, with an odds ratio (OR) of 0.974 and a 95% confidence interval (CI) ranging from 0.875 to 1.083 (*p* value of 0.629). Additionally, the *p* values for MR–Egger, weighted median, and simple mode all exceeded 0.05, confirming these results (Table 1; Figure 3). Figure S4 provides a forest plot that presents variant‐specific inverse variance estimates. The robustness of these findings was affirmed by the leave‐one‐out test, which is illustrated in Figure S5. Furthermore, Figure S6 shows a funnel plot that provides additional analysis of the association between Streptococcus and basal cell carcinoma.

**FIGURE 3:** Scatter plot of the causal association between Streptococcus and basal cell carcinoma.

Table 2 reveals no evidence of pleiotropy in the connection between Streptococcus and basal cell carcinoma [odds (intercept), 0.001; *p* = 0.912]. MR‐PRESSO analysis found no outliers (MR‐PRESSO global *p* value = 0.807). The *p* value from Cochran's Q test suggested the absence of heterogeneity in the analysis (Q = 5.136, *p* = 0.953).

### 3.3 Causal association of proteobacteria with basal cell carcinoma

According to the results of MR–Egger, IVW, simple mode, weighted mode, and weighted median, it can be inferred that there exists no causal association between Proteobacteria and basal cell carcinoma (IVW: OR = 1.113, 95% CI = 0.977–1.267, *p* = 0.106; MR‒Egger: OR = 1.111, *p* = 0.607; weighted mode: OR = 1.122, *p* = 0.203; simple mode: OR = 1.197, *p* = 0.244; weighted mode: OR = 1.184, *p* = 0.291) (Table 1; Figure 4). The forest plot in Figure S7 displays variant‐specific inverse variance estimates that emphasize that there is no possible causal connection between Proteobacteria and basal cell carcinoma. The robustness of these findings was validated by the leave‐one‐out test depicted in Figure S8. Furthermore, Figure S9 depicts a funnel plot delving deeper into the association between Proteobacteria and basal cell carcinoma.

**FIGURE 4:** Scatter plot of the causal association between proteobacteria and basal cell carcinoma.

As shown in Table 2, there was no indication of pleiotropy for the relationship between Proteobacteria and basal cell carcinoma [odds (intercept), 6.92e‐5; *p* = 0.995]. MR‐PRESSO analysis found no outliers (MR‐PRESSO global *p* value = 0.654). The *p* value of Cochran's Q did not reveal any heterogeneity, as indicated by a Q statistic of 6.975 and a *p* value of 0.639.

### 3.4 Causal association of Lachnospiraceae with basal cell carcinoma

Table 1 presents MR estimates derived from various methods employed to assess the causal influence of Lachnospiraceae on basal cell carcinoma. These estimates collectively suggested no genetic causal relationship between Lachnospiraceae and basal cell carcinoma (IVW: OR = 1.027, 95% CI = 0.899–1.173, *p* = 0.688; MR‒Egger: OR = 1.014, *p* = 0.933; Weighted median: OR = 0.991, *p* = 0.901; Simple mode: OR = 0.951, *p* = 0.682; Weighted mode: OR = 0.969, *p* = 0.768) (Table 1; Figure 5). Figure S10 shows a forest map that shows no potential causal link between Lachnospiraceae and BCC. The robustness of these results was confirmed by the leave‐one‐out test, which is presented in Figure S11. Additionally, Figure S12 presents a funnel plot investigating the causal association between Lachnospiraceae and basal cell carcinoma.

**FIGURE 5:** Scatter plot of the causal association between Lachnospiraceae and basal cell carcinoma.

As shown in Table 2, there was no indication of pleiotropy for the relationship between Lachnospiraceae and basal cell carcinoma [odds (intercept), 9e‐4; *p* = 0.935]. MR‐PRESSO analysis found no outliers (MR‐PRESSO global *p* value = 0.150). The *p* value obtained from Cochran's Q test indicated the absence of heterogeneity in the analysis, with a Q statistic of 26.001 and a *p* value of 0.125.

## 4 DISCUSSION

In this study, both GWAS data and a two‐sample MR analysis approach were employed to investigate the impacts of four specific GM on BCC. We found that Streptococcus, Bacteroides, Lachnospiraceae and Proteobacteria did not affect the occurrence of BCC from a genetic point of view. There are no studies that have documented a causal link between the gut microbiota and BCC. This study showed, from a genetic perspective, that Streptococcus, Bacteroides, Lachnospiraceae and Proteobacteria do not influence the development of BCC. However, it cannot be ruled out that these four kinds of GM may affect BCC through alternative mechanisms.

The skin and intestines serve as active and intricate immune and neuroendocrine organs. They are frequently exposed to the external environment and harbour diverse microbiota.^33^ Most studies have shown the tumour‐promoting effect of GM, but antitumour effects have also been observed.^34^ Cancer patients frequently experience disruptions in their gut microbiota due to treatments that impact the composition of and immunity related to these microbial communities.^35^ While the association between this ecological imbalance and BCC remains unclear, it has been investigated to a limited extent concerning cancer in general.^36^ Furthermore, our study revealed that the connection between GM and skin diseases can primarily be elucidated through the concept of the gut‐skin axis.^37^ The notion of the gut‐skin axis delineates the mutual relationship between the gut microbiota and the health of the skin. Several mechanisms, including inflammatory agents and the immune system, govern this relationship.^38^ In addition, Guo et al. also found evidence of gut‐skin axis through MR analysis, and they found a positive causal relationship between psoriasis and inflammatory bowel disease.^39^ Consequently, the connection between the gut microbiota and skin cancer can be examined from the perspective of the gut‐skin axis.

Bacteroides, as intestinal symbionts, fulfill various functions, such as shielding against pathogens and supplying nourishment to other gut microorganisms.^40^ In certain genetic disorders, Bacteroides might facilitate colonization of specific intestinal pathogens, potentially culminating in the development of particular cancer types.^41^ Another conceivable mechanism contributing to colon cancer involves the production of biofilms by certain Bacteroides strains.^42^ Previous research has underscored the significance of mucin‐type O‐polysaccharides in mediating their mutually advantageous effects and direct impact on the interaction between Bacteroides and host tissues.^43^ In general, glycosylation is a crucial contributor to the normal growth and differentiation of cells and tissues. Aberrant glycosylation, when it occurs, can lead to various disorders, with cancer being especially prominent among them.^44^ As an illustration, irregularities in mucin‐type O‐glycans have been linked to both colon and breast cancer.^44^, ^45^ However, the relationship between Bacteroides and BCC has not yet been reported. This study is the first to prove that Bacteroides does not affect the occurrence of BCC from a genetic point of view, but we cannot rule out that Bacteroides affects the occurrence of BCC in other ways.

Streptococcus, a common purulent gram‐positive coccus, is abundant in both the human gut and nasopharynx. It is primarily responsible for causing purulent inflammation and hypersensitivity disorders, among other conditions.^46^ Recent investigations have revealed that colorectal cancer exhibits a high abundance of Streptococcus within the intestinal microbiota. Additionally, there is an association between an elevated proportion of Streptococcus and the development of colorectal cancer.^47^, ^48^ *Streptococcus bovis* has been shown to promote the progression of precancerous lesions by activating pro‐inflammatory interleukin (IL)−8 production to promote overproliferation and abnormal colonic recess formation in mouse models.^49^ Furthermore, Yu et al. uncovered a connection between alterations in stool streptococcal composition and the occurrence of gastric cancer and liver metastasis. Streptococcus was identified as having the potential to serve as a predictive marker for gastric cancer.^46^ However, the precise pathogenic mechanism of Streptococcus remains obscure. Elevated levels of interleukin‐8 (IL‐8) and cyclooxygenase‐2 (COX2) and increased cell proliferation are among the factors that might contribute to its carcinogenic properties,^50^ though the exact pathogenic mechanism of Streptococcus remains elusive. Elevated levels of interleukin‐8 (IL‐8), heightened cell proliferation, and cyclooxygenase‐2 (COX2) might contribute to its potential to cause cancer.

Proteobacteria ranks among the most prevalent phylum in the human gut microbiota. As gram‐negative bacteria, they have the capability to generate lipopolysaccharide and facultative flagellin. These characteristics can spur inflammation and confer a specific level of pathogenic potential.^51^ Some studies have found that Proteobacteria members are also associated with cardiovascular disease, especially an increase in Proteobacteria, which is related to the occurrence of cardiovascular events in the general population.^52^ Additionally, it was observed that individuals with asthma have a higher abundance of Proteobacteria than healthy individuals.^53^, ^54^ There have been no prior reports on the association between Proteobacteria and skin cancer. This study, for the first time, establishes that Proteobacteria does not elevate the risk of BCC from a genetic perspective. However, further research is necessary to explore the underlying mechanisms.

Lachnospiraceae members colonise the intestinal tract from birth, and their relative richness increasing over the life of the host.^55^ While Lachnospiraceae members predominantly produce short‐chain fatty acids, various subsets within this family are linked to a range of both intestinal and extraintestinal disorders.^56^ Many studies have found that metabolic syndrome, obesity, diabetes, liver disease, chronic kidney disease and inflammatory bowel disease are all associated with Lachnospiraceae.^56^ Our research determined that, at the genetic level, there is no causal link between Lachnospiraceae and BCC.

This study is the first instance of employing MR methodology to substantiate that Streptococcus, Bacteroides, Lachnospiraceae and Proteobacteria do not affect the occurrence of BCC from a genetic point of view.

MR research can minimise the impact of internal confounding variables and avoid the conclusion deviation caused by reverse causality. Furthermore, our sensitivity analysis did not reveal any signs of multiplicity or heterogeneity, signifying the statistical robustness of our results. Nonetheless, our study is not without limitations. First, the data utilised in our research derive from European populations, potentially restricting the generalizability of our findings to other demographic groups. Second, our analysis solely examined the causal impacts of four specific gut microbiota types on BCC, implying that our results may not comprehensively represent the entirety of the gut microbiota's influence on BCC. Finally, our study found that four kinds of intestinal flora had no effect on BCC from a genetic point of view, but it could not be ruled out that these four kinds of GM affect BCC in other ways.

## 5 CONCLUSION

We found that Streptococcus, Bacteroides, Lachnospiraceae and Proteobacteria did not increase the incidence of BCC at the genetic level, which provides new insight for the study of intestinal flora and BCC. However, our findings do not negate the potential of a nongenetic association. Conducting broader research is essential to explore these potential connections.

## CONFLICT OF INTEREST STATEMENT

The authors declare no conflict of interest.

## ETHICS STATEMENT

There is no ethical statement here, because of all data downloaded from the Internet.

## Supporting information


**Supplementary Materials**: Supplemental Figure S1: Forest plot of the causal association between Bacteroides and Melanoma. Supplemental Figure S2: Leave‐one‐out test plot of the causal association between Bacteroides and Melanoma. Supplemental Figure S3: Funnel plot of the causal association between Bacteroides and Melanoma. Supplemental Figure S4: Forest plot of the causal association between Streptococcus and Melanoma. Supplemental Figure S5: Leave‐one‐out test plot of the causal association between Streptococcus and Melanoma. Supplemental Figure S6: Funnel plot of the causal association between Streptococcus and Melanoma. Supplemental Figure S7: Forest plot of the causal association between Proteobacteria and Melanoma. Supplemental Figure S9: Funnel plot of the causal association between Proteobacteria and Melanoma. Supplemental Figure S10: Forest plot of the causal association between Lachnospiraceae and Melanoma. Supplemental Figure S11: Leave‐one‐out test plot of the causal association between Lachnospiraceae and Melanoma. Supplemental Figure S12: Funnel plot of the causal association between Lachnospiraceae and Melanoma.

**Supplementary Materials**: Supplementary Table S1: SNPs information used in MR analysis of Bacteroides and Melanoma. Supplementary Table S2: SNPs information used in MR analysis of Streptococcus and Melanoma. Supplementary Table S3: SNPs information used in MR analysis of Proteobacteria and Melanoma. Supplementary Table S4: SNPs information used in MR analysis of Lachnospiraceae and Melanoma.

## Data Availability

Data used in the present study are all publicly available. The authors will provide the data upon reasonable request.
